The article "Predictive parameters for selection of electronic tissue compensation radiotherapy in early-stage breast cancer patients after breast-conserving surgery" was published in 2016. Journal: Oncotarget.

# Predictive parameters for selection of electronic tissue compensation radiotherapy in early-stage breast cancer patients after breast-conserving surgery

**DOI:** 10.18632/oncotarget.9054

**Published:** 2016-04-27

**Authors:** Yanbo Song, Miao Zhang, Lu Gan, Xiaopin Chen, Tao Zhang, Ning J. Yue, Sharad Goyal, Bruce Haffty, Guosheng Ren

**Affiliations:** ^1^ Department of Radiation Oncology, The First Affiliated Hospital of Chongqing Medical University, Chongqing, China; ^2^ Department of Radiation Oncology, Rutgers Cancer Institute of New Jersey, Rutgers Robert Wood Johnson Medical School, Rutgers The State University of New Jersey, New Brunswick, New Jersey, USA; ^3^ Chongqing Key Laboratory of Molecular Oncology and Epigenetics, The First Affiliated Hospital of Chongqing Medical University, Chongqing, China

**Keywords:** breast cancer, radiotherapy, 3DCRT, electronic tissue compensation, anatomic parameter

## Abstract

Electronic tissue compensation (eComp) is an external beam planning technique allowing user to manually generate dynamic beam fluence to produce more uniform or modulated dose distribution. In this study, we compared the effectiveness between conventional three-dimensional conformal radiotherapy (3DCRT) and eComp for whole breast irradiation. 3DCRT and eComp planning techniques were used to generate treatment plans for 60 whole breast patients, respectively. The planning goal was to cover 95% of the planning target volume (PTV) with 95% of the prescription dose while minimizing doses to lung, heart, and skin. Comparing to 3DCRT plans, on the average, eComp treatment planning process was about 7 minutes longer, but resulted in lower lung V_20Gy_, lower mean skin dose, with similar heart dose. The benefits were more pronounced for larger breast patients. Statistical analyses were performed between critical organ doses and patient anatomic features, i.e., central lung distance (CLD), maximal heart distance (MHD), maximal heart length (MHL) and breast separation (BS) to explore any correlations and planning method selection. It was found that to keep the lung V_20Gy_ lower than 20% and mean skin dose lower than 85% of the prescription dose, eComp was the preferred method for patients with more than 2.3 cm CLD or larger than 22.5 cm BS. The study results may be useful in providing a handy criterion in clinical practice allowing us to easily choose between different planning techniques to satisfy the planning goal with minimal increase in complexity and cost.

## INTRODUCTION

Breast cancer has the highest incidence rate (25.2%) and the highest mortality rate (14.9%) among all cancers in women [1, 2]. Whole breast radiation therapy after breast conserving surgery (BCS) is the standard of care for patients with early-stage breast cancer. Many studies have shown that radiation therapy (RT) could improve both loco-regional control and survival [3–7]. However, radiation toxicities to normal tissues affect the patients' quality of life (QOL). A recent meta-analysis study reported 14% and 42% incidence rates of clinical and radiological pneumonitis for patients having received 3DCRT for breast cancer [8]. Another study based on 35,000 breast cancer patients found the mortality rate from heart disease after radiation therapy is 3.2% [9]. In addition, the radiation induced skin complication is also common for breast radiation therapy patients [10–16]. Therefore, it is desirable to choose a radiotherapy planning and delivery technology to minimize the normal tissue toxicities and complications without compromising target dose coverage.

In clinical practice, 3DCRT is the conventional technique for whole breast irradiation. It features two tangentially arranged opposing beams covering the whole breast with static photon fluence. The primary goal of the whole breast radiotherapy planning is to design a treatment plan that can lead to uniform dose distribution within the target volume. However, it is inevitable that certain normal tissues fall inside the irradiated area, e.g., lung and heart, and they also receive certain levels of therapeutic dose. In order to spare the normal tissues as much as possible while keeping the similar target coverage, various technologies have been developed and introduced. eComp RT technique provided by Varian Eclipse treatment planning system (Varian Medical Systems, Palo Alto, CA) utilizes dynamic multileaf collimator (MLC) to generate dynamic beam fluence for an individual beam field. With the adjusted beam fluence, normal tissue can be spared while keeping the target uniformly covered in whole breast irradiation [17–19]. eComp is similar to the more familiarized field-in-field (FIF) technique, in terms of tissue compensation. However instead of manually generating individual field aperture to come up with a composited fluence map as FIF, eComp allows user to work on the beam fluence directly. The designed beam fluence will be automatically converted to deliverable MLC segments in the end.

The First Affiliated Hospital of Chongqing Medical University has been using eComp for whole breast irradiation since 2009. However, we observed the eComp plans are not always superior to 3DCRT plans in terms of normal tissue sparing. In this study, we compared the dosimetric characteristics between eComp and 3DCRT plans for our treated patients. With statistical analysis, we tried to identify the anatomic features that may potentially be used as indications of using the eComp technique over the conventional 3DCRT technique for the benefits of normal tissue sparing. Based on these results, we derived some predicting factors to help identifying whether a patient would be benefited from the eComp technique.

## RESULTS

### Planning comparison

A well trained dosimetrist designed all the plans. The average time to generate a 3DCRT plan was 28 minutes, and about 35 minutes for an eComp plan. The mean numbers of monitor units (MU) required to deliver the 3DCRT and eComp were 274 ± 82 MUs and 302 ± 56 MUs, respectively (*P* = 0.102).

Table 1 shows the dosimetric comparisons between the 3DCRT plans and their corresponding eComp plans. It is evident that the PTV coverage between 3DCRT and eComp plans was similar. eComp plans delivered lower doses to ipsilateral lung and skin in comparison to their corresponding 3DCRT plans. However, no substantial difference was found in heart, liver, contralateral breast and contralateral lung doses between the two planning techniques. As examples, Figure 1 and Figure 2 show that the lung V_20Gy_ and the skin volumes received more than 100% prescription dose are lower in eComp plans than those in their corresponding 3DCRT plans.

**Table 1:** Comparison of PTV and OARs doses between 3DCRT and eComp

Metric	3DCRT	eComp	*P*-value
PTV			
D_mean_(Gy)	52.8 ± 0.7	51.6 ± 0.2	0.441
D_max_(Gy)	55.2 ± 0.2	53.8 ± 0.7	0.052
D_95_(Gy)	47.5 ± 0.7	48.7 ± 1.1	0.103
HI	0.51 ± 0.12	0.62 ± 0.13	0.070
CI	0.47 ± 0.22	0.49 ± 0.19	0.213
Ipsilateral Lung			
V_5_ (%)	32.3 ± 1.3	31.6 ± 2.4	0.033
V_10_ (%)	28.1 ± 1.8	26.7 ± 0.5	0.027
V_20_ (%)	16.8 ± 4.2	12.9 ± 2.1	0.000
V_30_ (%)	13.2 ± 1.4	12.6 ± 1.7	0.021
V_40_ (%)	11.3 ± 1.0	10.5 ± 1.5	0.131
D_mean_(Gy)	9.2 ± 2.3	7.7 ± 1.6	0.000
Heart			
V_20_ (%)	32.4 ± 1.3	30.9 ± 0.8	0.054
V_30_ (%)	28.7 ± 1.8	26.5 ± 0.5	0.271
V_40_ (%)	17.1 ± 1.8	14.9 ± 2.2	0.135
D_mean_(Gy)	4.6 ± 2.5	4.7 ± 2.7	0.209
Skin			
V_30_ (%)	32.4 ± 1.3	30.8 ± 1.6	0.030
V_40_ (%)	28.5 ± 1.8	26.9 ± 0.5	0.037
V_50_ (%)	17.2 ± 0.8	14.4 ± 1.2	0.024
D_mean_(Gy)	40.6 ± 1.6	39.5 ± 1.4	0.001
Liver D_mean_(Gy)	0.7 ± 0.3	0.8 ± 0.3	0.513
Contralateral Breast D_mean_(Gy)	1.4 ± 0.5	1.3 ± 0.7	0.438
Contralateral Lung D_mean_(Gy)	0.8 ± 0.3	0.9 ± 0.2	0.376
MU	274 ± 82	302 ± 56	0.102
Processing Time (min)	28 ± 3	37 ± 2	0.071

Abbreviations: 3DCRT = three-dimensional conformal radiotherapy; eComp = electronic tissue compensation; HI = homogeneity index; CI = conformity index; MU = monitor unit.

**Figure 1:** Comparison of isodose line of lung V_20Gy_ (green line) (**A**) The coverages of 95% isodose line (cyan) for PTV (red) were similar between techniques. More lung volume involved in the isodose line of 20 Gy in 3DCRT plan from one patient. (**B**) Comparing to 3DCRT, less lung volume involved in the isodose line of 20 Gy in eComp plan for the same patient.

**Figure 2:** Comparison of skin volumes received more than 100% prescription dose (PD) in three views (**A-1, 2, 3**) The skin volumes received more than 100% PD from axial, sagittal and coronal views in 3DCRT plan from one patient. (**B-1, 2, 3**) The volume of corresponding dose in eComp plan is much smaller than those in 3DCRT plan.

### Correlations between the anatomic and dosimetric parameters

Figure 3 shows that the ipsilateral lung V_20Gy_ had a linear correlation to CLD in both 3DCRT (R^2^ = 0.775) and eComp (R^2^ = 0.642) plans. For any given patient, the ipsilateral lung V_20Gy_ would be higher in a 3DCRT plan than an eComp plan. If the lung V_20Gy_ was limited to be less than 20%, the 3DCRT plan could only be used for patients with CLD less than 2.3 cm. On the other hand, the eComp technique could be used to generate plans on patients with CLD up to 3.5 cm with V_20Gy_ being still less than 20%.

**Figure 3:** The correlation between ipsilateral lung V_20_ and CLD for 3DCRT and eComp The ipsilateral lung V_20_ increases linearly with the CLD for both 3DCRT and eComp. When CLD increases to 2.3 cm, the ipsilateral lung V_20_ will tend to exceed 20% of lung volume for 3DCRT, which predicts the need for eComp RT technique.

MHD and MHL also had linear correlation with the mean heart dose for both techniques as shown in Figures 4, 5. The similar slopes between the eComp and 3DCRT plans demonstrated that the mean heart dose differences were small between those two techniques.

**Figure 4:** The correlation between mean heart dose and MHD for 3DCRT and eComp The mean heart dose increases linearly with the MHD for both 3DCRT and eComp. The similar slopes between the eComp and 3DCRT plans demonstrated the mean heart dose differences were small between those two techniques.

**Figure 5:** The correlation between mean heart dose and MHL for 3DCRT and eComp The mean heart dose correlated linearly with the MHL both in 3DCRT and eComp. The similar slopes between the eComp and 3DCRT plans showed the mean heart dose differences were small between those two techniques.

Figure 6 shows a loose but positive correlation between BS and the mean skin dose. The correlation coefficients (R^2^) for 3DCRT and eComp plans were 0.473 and 0.432, respectively. The trend of the regression lines show eComp technique was more likely to generate plans with lower skin dose comparing to 3DCRT for larger breast patients. Ifthe mean skin dose limit was to be less than 85% of the prescription dose as followed in our institution, 3DCRT could be only planned on patients with 22.5 cm or less breast separation whereas eComp could be used for patients with the breast separation up to 29.6 cm.

**Figure 6:** The correlation between mean skin dose and BS for 3DCRT and eComp When BS exceeds 2.2 cm, in 3DCRT, the mean skin dose would higher than the dosimetry constraint criteria (D_mean_ ≤ 85% of target dose). Hence, BS = 2.3 cm may be considered as a cutoff point to decide when the eComp should be used to decrease the skin dose.

## DISCUSSION

The dosimetric comparisons demonstrated patients could benefit from eComp technique over the conventional 3DCRT technique in the whole breast irradiations. However, considering the extra effort to manually tweak the beam fluence to generate an eComp plan, it is not cost effective to plan every patient with eComp if a simple yet effective 3DCRT plan can be generated. “Which planning technique to choose for a given patient?” should be the question to be answered in the first place. In our work, the regression analysis between normal tissue doses and patient anatomic parameters provided some guidance on this question. Figure 3 and Figure 6 can be used as the worksheets to determine the techniques once the patient's anatomic features were measured from the simulation CT. For example, based on the measurement on simulation CT, a patient is found to have CLD of 3 cm and BS of 25 cm; the planning goal is to keep the lung V_20Gy_ less than 20% and the mean skin dose less than 42 Gy; according to Figure 3 and Figure 6, if 3DCRT is used, the lung V_20Gy_ and the mean skin dose would be 25% and 43 Gy. On the other hand, the corresponding dosimetric values for an eComp plan would be only 16% and 41 Gy. In that case, an eComp plan should be selected over 3DCRT. However, if it is found that CLD is only 2 cm and BS 20 cm, a 3DCRT plan would yield 18% lung V_20Gy_ and 41 Gy mean skin dose. Then, 3DCRT should be an effective choice for the patient.

In our study, heart dose was analyzed for left-sided breast patients only. The mean heart dose was found to linearly increase with the MHL and MHD. However, the differences between 3DCRT and eComp were negligible. As shown in Table 1, the mean heart dose was less than 5 Gy in both techniques. Given the fact that the heart dose constraint is easy to meet, it may not need to be taken into consideration in deciding which of the two techniques is preferred.

In photon based external beam therapy, 3DCRT technique utilizes simple beam modifiers, such as wedges, to modify beam fluence. It has the fewest degrees of freedom to modulate the dose delivery patterns. At the other extreme is the intensity-modulated radiation therapy (IMRT), which uses inverse planning and dynamic multileaf collimator (MLC) to generate plans with optimized dynamic fluence [20, 21]. However, the use of IMRT will substantially increase the cost to patients and workload to physicians, physicists and dosimetrists [22, 23]. It may also increase the machine output MUs in delivering the beams, and may lead to undesired late effects (e.g., secondary cancers) to patients. eComp technique lies somewhere in between 3DCRT and IMRT, in terms of planning and delivery complexity. Based on our study, its use can reduce the normal tissue doses in the whole breast irradiations with acceptable increases in complexity and cost.

In our institution, till the time this research study was completed, we had not have treated any very large and pendulous breast patients. Since most of our patient had relative small separations, only 6 MV photon beams were used in treatment. For large size breast patients, the use of higher energy photon beam (e.g., 15 MV) would be helpful to achieve better dose uniformity, but at the expense of patient being exposed to whole body neutron dose. Since the physical features of percent depth dose of higher photon beam are similar to those of 6 MV beam except for degree of penetration, we anticipate that the findings from this study should be valid for those situations with 15 MV photon beams, but with different cutoff values. However, additional studies are needed to prove it.

In this study, V_20_ for lung, mean dose for heart and skin mean doses were used to evaluate the toxicities to the 3 normal organs commonly involved in the breast cancer treatment. We also analyzed other parameters for lung, heart and skin in the Result section and in Table 1. The analysis showed that there are minimal differences between eComp and 3DCRT for the other parameters. In addition, according to literatures [8, 9, 37, 44] and protocols of our institution, those 3 quantities were generally considered as the determining factors in the normal tissue toxicities. In order to keep the consistency and to reduce plan differences caused by different planners, we decided that all plans were done by a single well-trained dosimetrist. Although this approach reduces the planner difference, it may also lead to results embedded with planer's bias. Therefore, the results of this study can only be used as general guidelines rather than strict rules.

We recognize that the number of cases included in this study is still relatively small to draw more definitive conclusions on using the anatomic parameters to predict the more appropriate planning and delivery technique in whole breast irradiations. It is noticed that for all the fitting exercises, except for the lung V_20_ plot, other data series were mixed and scattered around the fitting line with a small *R* value. Hence the results may only be served as a general guideline in clinic. A further study to validate our current findings in a larger cohort is warranted. In addition, this study only included the early-stage breast cancer patients who did not need regional lymph nodes irradiation. Due to this limitation, caution should be taken when generalizing the current results to the patient groups requiring nodal regional radiotherapy.

## MATERIALS AND METHODS

### Patient selection and image acquisition

After approval from the Institutional Review Board (IRB), a total of 60 patients with 26 left-sided and 34 right-sided breast cancer patients were reviewed and used in the study retrospectively. All patients had stage 0, I or II unilateral histological-confirmed breast cancer after BCS. The mean age of these patients was 48 years old ranging from 32 to 58. The simulations were performed on a GE CT scanner (GE Medical Systems, Milwaukee, WI). Patients were positioned supinely on a breast board with ipsilateral arm extended above the head and the head turned to the contralateral side. The scanned region extended from the mid-neck to 5 cm below the inferior border of the breast with 2.5 mm slice thickness.

### Definition of the target volumes and organs at risk (OAR)

The clinical target volume (CTV) was defined as the entire breast tissue, based on skin contour and palpation, and was 3 mm inside the skin surface. The planning target volume (PTV) was generated by expanding the CTV 5 mm in all directions, except towards the skin surface where no margin was added. The mean planning target volume (PTV) and breast separation were 528 cc (from 215 cc to 1260 cc) and 23.1 cm (from 19.2 cm to 26.8 cm), respectively.

Following the OAR contouring atlases of RTOG 1106 [24, 25], the heart, ipsilateral and contralateral lungs, skin, liver and contralateral breast were contoured as the normal tissues. The heart was contoured only for 26 left-sided patients. The superior aspect started at the level of the inferior aspect of the pulmonary artery passing the midline and extended inferiorly to the cardiac apex. Ipsilateral and contralateral lungs were contoured separately using pulmonary windows. The skin was delineated as from the body surface to 3 mm inward. The liver was contoured only for patients with right-sided breast cancer. The contralateral breast was manually delineated.

### Treatment planning

Varian Eclipse treatment planning system (version 10.0, Varian Medical System, Palo Alto, CA) was used to generate 3DCRT and eComp plans for each patient, respectively. The prescription dose was 50 Gy in 25 fractions for all patients followed by a 10 Gy boost with electron. The electron boost was not considered in the comparison. In all plans, the primary dose coverage goal was 95% of PTV receiving at least 95% of the prescribed dose with the maximum dose less than 110% of the prescription dose.

### 3DCRT plans

3DCRT plans consisted of two opposing tangential 6MV photon beams. MLC were formed to shield heart and lung as needed while providing adequate dose coverage to the target volume. Beam wedges were used as needed to meet the dose uniformity criteria.

### eComp plans

eComp plans used the identical beam arrangements as the corresponding 3DCRT plans. Instead of using wedges, the tissue compensation function was employed to create a dynamic MLC fluence map. The fluence map was edited manually to achieve a desired dose distribution. Then, the optimum fluence map was extended beyond the patient surface by the skin flash tool provided in Eclipse then converted to a deliverable fluence based on the specific characterization of the dynamic MLC (Figure 7).

**Figure 7:** Electronic tissue compensation was employed to create a dynamic MLC fluence map The optimum fluence map was extended beyond the patient surface by the skin flash tool provided in Eclipse then converted to a deliverable fluence based on the specific characterization of the dynamic MLC.

### Dose-volume parameters

PTV D_95_ (the dose delivered to 95% of the volume), D_max_ (the maximum dose) and D_min_ (the minimum dose), homogeneity index (HI) and conformity index (CI) were calculated. The following equations were used to calculate HI [26] and CI [27].

$$\text{HI}=({\text{D}}_{2\%}-{\text{D}}_{98\%})/{\text{D}}_{50\%}$$

where D_2%_, D_98%_ and D_50%_ are the minimum absorbed doses covering 2%, 98% and 50% of the volume of the PTV.

$$\text{CI}=({\text{V}}_{\text{PTV}}/{\text{TV}}_{\text{PV}})/({\text{TV}}_{\text{PV}}/{\text{V}}_{\text{TV}})$$

where V_PTV_ is the volume of PTV, TV_PV_ is the volume of PTV covered by the prescription dose, and V_TV_ is the volume covered by the prescription dose.

The mean dose and other dose volume parameters, e.g., D_mean_, V_5Gy_, V_10Gy_, V_20Gy_ to V_50Gy_, are calculated also for heart, lung and skin.

### Anatomic parameters

A number of studies have utilized anatomic parameters to evaluate the doses to the organs at risk(OAR) in whole breast irradiation using 3DCRT and other modified IMRT [13, 28–36]. In order to explore the selection criteria for patients who will benefit from eComp based treatments, the anatomic features including breast separation (BS), central lung distance (CLD), maximal heart distance (MHD) and maximal heart length (MHL)were measured in a DRR view of one of the fields (Figure 8). The BS was defined as the distance between entry points of two opposing beams on the central plane. The CLD was defined as the maximum perpendicular distance from the posterior edge of the tangential field to the posterior part of the anterior chest wall in the middle of the field. The MHD and the MHL were defined as the maximal width and length of the heart contour intercepted by the posterior boarder of the tangential fields.

**Figure 8:** Anatomic parameters **(A) PTV was contoured in red.** The breast separation (BS) is the distance between entry points of two opposing beams on the central plane. The central lung distance (CLD) is the perpendicular distance from chest wall to the posterior boarder of the tangential fields. (**B**) The heart was contoured in orange. The maximal heart distance (MHD) and the maximal heart length (MHL) are the width and length of the heart contour intercepted by the posterior boarder of the tangential fields.

### Statistical analysis

A paired *t* test or signed rank test was applied to compare the average differences in the dose-volume parameters between the two techniques. The level of two-tailed statistical significance was set at 0.05.

To test the impact of the anatomic parameters on organ doses, linear regression analyses were performed between each of the anatomic parameters and the selected dose-volume parameters of the related normal tissues. The regression pairs were: ipsilateral lung V_20Gy_ with CLD, mean heart dose with MHD and MHL, respectively, and mean skin dose with BS. The correlation between heart dose-volume parameters and anatomic features was analyzed only for left-sided patients. Those dose-volume parameters were selected due to the fact that they are generally considered as the determining factors on the normal tissue toxicities [8, 30, 35, 37–44].

## CONCLUSIONS

For whole breast irradiation, eComp plans resulted in lower lung V_20Gy_ and lower mean skin dose than the traditional 3DCRT plans. The benefit was more prominent for patient with large CLD and BS. The CLD and BS were identified as two predicting factors to determine which planning technique to use for a given breast patient.
